# Toll-Like Receptor Ligands Induce Human T Cell Activation and Death, a Model for HIV Pathogenesis

**DOI:** 10.1371/journal.pone.0001915

**Published:** 2008-04-02

**Authors:** Nicholas Funderburg, Angel A. Luciano, Wei Jiang, Benigno Rodriguez, Scott F. Sieg, Michael M. Lederman

**Affiliations:** 1 Department of Molecular Biology and Microbiology, Case Western Reserve University, Cleveland, Ohio, United States of America; 2 Division of Neonatology, Department of Pediatrics, Rainbow Babies and Children's Hospital, Cleveland, Ohio, United States of America; 3 Department of Medicine, Center for AIDS Research, Case Western Reserve University, University Hospitals/Case Medical Center, Cleveland, Ohio, United States of America; New York University School of Medicine, United States of America

## Abstract

**Background:**

Recently, heightened systemic translocation of microbial products was found in persons with chronic HIV infection and this was linked to immune activation and CD4^+^ T cell homeostasis.

**Methodology:**

We examined here the effects of microbial Toll-like receptor (TLR) ligands on T cell activation *in vitro*.

**Conclusions/Findings:**

We show that exposure to TLR ligands results in activation of memory and effector CD4^+^ and CD8^+^ T cells. After exposure to each of 8 different ligands that activate TLRs 2, 3, 4, 5, 7, 8, and 9, CD8^+^ T cells are activated and gain expression of the C type lectin CD69 that may promote their retention in lymphoid tissues. In contrast, CD4^+^ T cells rarely increase CD69 expression but instead enter cell cycle. Despite activation and cell cycle entry, CD4^+^ T cells divide poorly and instead, disproportionately undergo activation-induced cell death. Systemic exposure to TLR agonists may therefore increase immune activation, effector cell sequestration in lymphoid tissues and T cell turnover. These events may contribute to the pathogenesis of immune dysfunction and CD4+ T cell losses in chronic infection with the human immunodeficiency virus.

## Introduction

Microbial challenge is recognized by cells of the innate immune system through the interactions of conserved microbial structures with a family of type 1 transmembrane receptors called Toll-like receptors (TLRs). To date, 10 members of the TLR family, that differ in ligand specificities and expression patterns, have been described in humans [1], [2]. Recently, translocation of microbial products from the gut has been implicated as important in the pathogenesis of immune activation in chronic HIV infection [3]. Increased blood levels of the TLR4 ligand lipopolysaccharide (LPS) have been found in chronic HIV infection and these levels correlate directly with immune activation and inversely with CD4^+^ T cell restoration after antiviral therapies. Moreover, LPS levels were increased in the blood of pathogenic (rhesus) SIV infection but not in non-pathogenic SIV infection of sooty mangabeys that characteristically do not experience immune activation and high T cell turnover during chronic infection [4]. We show here that *in vitro* exposure to microbial TLR ligands promotes selective activation and death, especially of memory and effector T cells that may contribute to the pathogenesis of immune deficiency in chronic HIV infection.

## Results

### TLR ligands can induce early activation marker expression on CD4^+^ and CD8^+^ T cells

To evaluate responsiveness of T cell populations to TLR stimulation, whole PBMCs were cultured in medium alone, or in medium supplemented with a TLR ligand. After overnight culture with ligands for TLR 3, 4, 5, and 9, expression of CD38 (but not HLA-DR) was induced on both CD4^+^ and CD8^+^ T lymphocytes (Figure 1)

**Figure 1:** Stimulation of peripheral blood cells by Toll-like Receptor ligands increases expression of CD38 on CD4+ and CD8+ T lymphocytes. PBMC were cultured overnight in medium alone, or stimulated with individual TLR ligands (Poly-I:C, LPS, Flagellin, or CpG DNA) or with plate-bound anti-CD3 antibody. Expression of CD38 and HLA-DR was monitored by flow cytometry among: (A) CD4+ T cells and (B) CD8+ T cells. Percentages of cells expressing each marker are shown. This experiment is representative of 5.

### Central memory and effector/memory CD4^+^T cells enter cell cycle while memory/effector CD8^+^ T cells express high levels of CD69 after exposure to TLR ligands

We next examined surface expression of CD69, a C type lectin implicated in the retention of activated T cells within lymph nodes [5], [6], and intracellular expression of Ki-67, a marker of cell cycle entry. After 7 days' cultivation with each TLR ligand, CD8^+^ T cells were induced to express high levels of CD69, and CD4^+^ T cells entered cell cycle (Figures 2A, 2B). These two pathways of cellular activation were relatively selective for the different T cell subpopulations as activated CD4^+^ T cells only increased CD69 expression significantly in response to Flagellin A and poly U stimulation and otherwise were rarely found to express CD69 at any time after stimulation (D1, D3, D5, or D7, not shown). On the other hand, activated CD8^+^ T cells entered cell cycle less frequently than did the activated CD4+ T cells and only in the presence of certain ligands (PGN, poly I:C, Flagellin A, Imiquimod, and CpG DNA) did treated cells enter cycle more frequently than did cells cultured in medium alone. Each TLR ligand was tested at multiple concentrations (not shown) and results are shown using an optimal concentration for each agonist. Interestingly, maturation phenotype predicted the magnitude of response such that in response to most ligands, central memory and effector memory CD4+ T cells more often entered cell cycle than did naïve CD4+ T cells and among CD8+ T cells, effector memory cells tended to have the greatest frequency of CD69 expression. (Figure 3A–D).

**Figure 2:** TLR ligands induce high level CD69 expression on CD8+ T cells and Ki- 67 expression in CD4+ T cells. Intracellular expression of Ki-67 (A) and surface expression of CD69 (B) were monitored after 7 days of cell culture in medium or with the stimuli as indicated. Bars represent means and the lines standard errors of the mean (SEM) of 15 separate experiments using PBMC of healthy controls. Black boxes = CD4+ T cells and gray boxes = CD8+ T cells. * = nominally significantly different (p<0.05 by Wilcoxon Sign Rank test when compared to results obtained in medium alone.

**Figure 3:** TLR ligands preferentially activate CD4+ central memory and effector memory T cells and CD8+ effector memory T cells. Intracellular Ki-67 expression (3A, 3C) and cell surface CD69 (3B, 3D) were analyzed after 7 days' incubation of PBMC in medium alone, or in medium supplemented with plate bound anti-CD3 antibodies, or the indicated TLR ligand. Figures 3A and B are representative results among phenotypically defined naïve (CD45RA^+^CD45RO^−^CCR7^+^), central memory (CD45RA^−^CD45RO^+^CCR7^+^), and effector memory (CD45RA^−^CD45RO^+^CCR7^−^) CD4^+^ and CD8^+^ T cells. Values represent percentages of cells staining for Ki-67 or CD69. Figures 3C and 3D reflect the mean data from 15 separate experiments. Values nominally significantly different from medium alone values (Wilcoxon Sign Rank Test) are shown with an asterisk.

### The TLR 3 ligand poly I:C can activate T cells directly and despite expression of TLR 5, purified T cells require an intermediary cell for activation by the TLR 5 ligand flagellin

We were able to confirm expression of TLR-3 and TLR-5 in circulating T lymphocytes while expression of TLR2 was not convincing (Figure 4). Expression of these TLRs on both CD4^+^ and CD8^+^ phenotypically defined naïve (CD45RA^+^CD45RO^−^CCR7^+^) and memory (CD45RA^−^CD45RO+) T cell subsets mirrored their expression in the unseparated T cell populations (not shown). Exposure to the TLR 3 ligand poly I:C could induce CD38 expression directly on purified T cells (Figure 4B). On the other hand, while T cells within PBMC preparations could be activated to express CD38 after exposure to the TLR5 ligand flagellin, purified T cells were not; nor could they be induced to express CD38 through transwell exposure to soluble products of flagellin-stimulated PBMC (Figure 4B).

**Figure 4:** Toll-like receptors 3 and 5 are expressed by a subset of T cells, but expression is not always sufficient for activation by TLR ligands. (A) Whole PBMCs were isolated from healthy donors and expression of TLRs 2, 3, and 5 were evaluated by flow cytometry on gated CD3+ T cells. (B) Whole PBMCs, purified T cells (>95% CD3^+^), or purified T cells separated from whole PBMCs by a transwell, were cultured in medium alone, or in medium supplemented with plate bound anti-CD3, poly I:C or flagellin A. Expression of CD38 on memory (CD45RO^+^CD45RA^−^) CD4^+^ T cells was assessed by flow cytometry following overnight culture. Dotplots shown are representative of 8 separate experiments.

### TLR ligand exposure preferentially induces CD4^+^ T lymphocyte apoptosis

TLR ligation is thought to play a role in B cell homeostasis by promoting expansion and survival of both memory [7] and naïve [8] B lymphocytes. We therefore examined the effects of TLR ligands on the *in vitro* expansion of CD4^+^ and CD8^+^ T cells after staining with CFSE (Figure 5). Despite substantial movement of CD4^+^ T cells into cycle after exposure to TLR ligands (Figure 2A), there was little dilution of dye that would reflect cell division. In contrast, there was substantial evidence of cell death as reflected in Annexin V binding. As CD8^+^ T cells infrequently entered cell cycle after TLR ligation, a failure of cellular proliferation was not surprising. Nonetheless, even among CD8^+^ T cells, exposure to TLR ligands resulted in more Annexin V binding than was seen among cells cultured in medium alone.

**Figure 5:** Activation as a result of TLR ligand exposure preferentially induces T cell death especially among CD4+ T cells. PBMCs were labeled with CFSE and incubated for 6 days in the presence of anti-CD3 antibody, medium alone or TLR ligands alone (PGN, poly-I:C, LPS (10 or 20 ng/ml), Flagellin A, Flagellin B or imiquimod). After 6 days of incubation, the CD4^+^ and CD8^+^ T cells were examined for dilution of CFSE dye and for binding of Annexin V. Numbers in right upper corners represent percentage of Annexin V-binding cells. Numbers in the left lower corner represent percentage of cells that diluted dye without Annexin-V binding. This experiment is representative of three separate experiments.

## Discussion

Toll-like receptors play a critical role in early recognition of potential pathogens [2], [9]. Broadly expressed by epithelial cells, phagocytic, and antigen- presenting cells, TLRs are critical sensors for innate immune defenses, allowing rapid detection and responsiveness to elements expressed by a wide range of microbes. There is increasing recognition that the innate and adaptive defense systems are linked. Thus, TLR ligation results in production of inflammatory cytokines and increased expression of co-stimulatory molecules and class I and II MHC antigens, leading to more a more effective presentation of peptides to promote T cell activation and expansion [2], [9], [10]. The recent demonstration of selected TLR RNAs and protein in T cells suggested that these ancient receptors also may have a direct role in the maturation or expansion of the adaptive cellular immune response [1]. In these experiments, we therefore asked if TLR ligand exposure could promote T cell activation. We find that even in the absence of high affinity T cell receptor engagement, TLR agonists can induce activation of CD4^+^ and CD8^+^ T lymphocytes. Shortly after exposure, both CD4^+^ and CD8^+^ T cells show increased surface expression of the activation-related multifunctional ectoenzyme CD38 that is highly expressed on activated T lymphocytes in HIV infection and is a strong predictor of disease progression therein [11]–[14]. After longer term cultivation, CD4^+^ and CD8^+^ T cells showed distinctly different pathways of activation. CD4^+^ T cells were induced to enter cell cycle and rarely expressed the C-type lectin CD69 on the cell surface. In contrast, CD8^+^ T cells were activated to express CD69, and were less frequently induced to enter cell cycle. Importantly, among CD4+ T cells, naïve cells were less frequently activated than were memory and effector populations except in response to the TLR 3 ligand polyI:C that activates T cells directly. Among CD8+ T cells, cells of the effector memory phenotype were most activated to express CD69 by TLR agonist exposure while activation of central memory and naïve phenotype cells was generally less dramatic although exposure to the TLR 3 agonist polyI:C and to the TLR 7 agonist poly U resulted in substantial activation of all CD8+ T cell maturation phenotypes.

Interestingly, despite the clear demonstration of TLR5 on circulating T cells, purified T lymphocyte populations were not responsive to the TLR5 ligand flagellin nor were they responsive to soluble products of PBMC preparations in which flagellin responses were demonstrable. Thus an intermediary contact with a TLR 5-expressing accessory cell is likely necessary to promote T cell activation in response to this ligand. On the other hand, purified T cells could be activated directly in response to the TLR 3 ligand poly I:C. While it is possible that low level contamination of these purified T cell populations with TLR-bearing accessory cells may have contributed to the T cell activation by poly I:C, it should be noted that these same T cell preparations were sufficiently depleted of accessory cells to remain unaffected by anti-CD3 stimulation. Thus, for at least one TLR ligand, poly I:C, T cells may be activated directly; for flagellin, despite clear expression of TLR5, T cells are not activated directly, but require the presence of accessory cells. Thus, for some ligands like flagellin, TLR expression on T cells is not sufficient to promote T cell activation. Whether TLR expression is necessary for T cells to be activated in response to TLR ligands is not clear but the very low levels of certain TLR mRNAs and protein found among purified T cells [1], [10], [15], [16] and the substantial T cell activation in response to many TLR ligands that bear poor relationships to TLR expression levels suggests that T cell expression of these receptors may not be necessary for responses to certain of these TLR agonists. .

Purified human CD4^+^ T lymphocytes proliferate and secrete cytokines in response to flagellin or R848, when a secondary signal such as anti-CD3 or IL-2 is also provided [16]. Regulatory T cell function is enhanced and levels of the transcriptional regulator FOXP3 are increased after exposure to flagellin and TCR stimulation [15]. Though direct exposure of human T cells to LPS does not induce proliferation or cytokine secretion; phosphorylation of p38 and Pyk-2 and altered chemotactic responses to stromal cell derived factor 1α (SDF-1α) are demonstrable [17]. Our studies are the first to describe the consistent and differential responsiveness of CD4^+^ and CD8^+^ T maturation subsets after stimulation with a broad panel of TLR ligands. Activation of T cells by TLR ligands was especially demonstrable among phenotypically defined memory or memory/effector cells, as naïve cells were far less responsive to TLR agonist exposure. Thus, exposure to TLR ligands at sites of microbial invasion may selectively enhance activation of memory and effector T cells that are concurrently engaged through their TCRs or perhaps even via bystander cytokine costimulation.

There is increasing evidence to suggest that T cell activation by TLR ligands also may play an important role in HIV disease pathogenesis. Recently, RNA sequences derived from the HIV-1 genome have been shown to induce activation via interactions with TLR 7/8 [18], [19] and this interaction may activate T cell populations indirectly [20]. Very recently, we found high levels of bacterial LPS in the plasmas of persons with chronic HIV infection [3]. Levels of LPS were correlated with indices of T cell activation and with plasma levels of interferon-alpha and predicted inversely the magnitude of CD4+ T cell restoration after application of HAART. These findings suggest that the gut barrier to systemic translocation of a variety of commensal microbial elements is perturbed in chronic HIV infection as LPS does not characteristically induce alpha interferon expression. The importance of this model in HIV disease pathogenesis is suggested by the demonstration that in the pathogenic (rhesus) model of SIV infection, LPS levels were increased in infected animals, while in the non-pathogenic (sooty mangabey) model, SIV infection did not increase plasma LPS levels [3]. More recently, we have found increases in circulating levels of bacterial DNAs in chronic HIV infection and these bacterial DNA levels also were correlated with indices of immune activation and cellular restoration after application of antiviral therapies (unpublished data).

Our data may provide insights as to how systemic exposure to a number of microbial TLR agonists drives immune activation and disease pathogenesis in HIV infection. Secondary lymph nodes in chronic HIV infection tend to be enriched for effector CD8+ T cells of numerous specificities that are ordinarily relatively excluded from these sites [21]–[25]. Induction of CD69 by type I interferons has been associated with intracytoplasmic retention of the sphingosine-1 phosphate (S1P) receptor S1P1 that facilitates exit of activated T cells from lymphoid tissues [6]. Thus, induction of CD69 expression by TLR ligand exposure may thereby result in inappropriate sequestration of activated CD8+ EM T cells in lymphoid tissue where they contribute to the lymphadenopathy [26] and inflammatory cytokine storm that characterizes HIV infection [24], [27]. In earlier work we [28] and others [29], [30] have found high frequencies of circulating S phase CM T cells in HIV and SIV infections respectively. These cells turn over rapidly in untreated infection [29]–[32]. We show here that T cell activation induced by TLR agonist exposure results in activation of CD4+ CM and EM T cells to enter cell cycle and a heightened tendency for the activated T cells to die. This is most apparent in the CD4^+^ T cell population. Although these cells progress into S phase (not shown), there is minimal evidence of complete cell division, as is seen after TCR stimulation (Figure 5). Likewise, though movement of cells into cell cycle is often associated with some level of cell death, this is disproportionately increased in cells activated in the presence of TLR agonists. Among CD8^+^ T cells, even though they are infrequently activated by TLR ligand exposure to enter cell cycle, they also tend to become apoptotic after activation, though less frequently than CD4^+^ T cells do.

In summary, in vitro exposure of peripheral blood mononuclear cells to a variety of microbial TLR agonists results in activation of T cells predominantly of central memory and effector memory phenotype. CD8+ EM cells are activated to express CD69 that may promote their retention in secondary lymphoid tissues while CD4+ CM and EM T cells are activated to enter cell cycle and to die. We provide here an indication of how systemic exposure to microbial TLR agonists that include both HIV RNAs and a variety of bacterial elements translocated from the damaged gut may drive T cell activation and cell death in chronic HIV infection.

## Materials and Methods

### Subjects

These studies were approved by the Institutional Review Board of University Hospitals/Case Medical Center. Blood samples were obtained from 20 healthy donors.

### Cells

Blood was collected in heparin-coated tubes and peripheral blood mononuclear cells (PBMCs) were isolated by centrifugation over Ficoll-Histopaque. The culture medium consisted of RPMI 1640 (Bio Whittaker, Walkersville, MD) supplemented with 50U/ml penicillin, 50 µg/ml penicillin/streptomycin, 2mM L-glutamine (Bio Whittaker) and either 10% fetal bovine serum (Gemini Bioproducts, Woodland, CA) or 10% Human AB serum (Gemini Bioproducts). Monocytes and T cells were negatively selected by immunoaffinity using MACS isolation kits (Monocyte Isolation kit II and the Pan T cell kit, respectively) (Miltenyi Biotec, Bergisch Gladbach, Germany). Monocytes and T cells were evaluated for purity based on CD14 or CD3 expression and were 85–90% and 95–98% pure, respectively. Transwell experiments were performed using membrane inserts containing 0.4 µM pores (Corning Incorporated, Corning, NY)

### Cell culture

PBMCs were stimulated with plate bound-anti-CD3 monoclonal antibodies (BD Pharmigen, San Diego, CA; 10 µg/ml) or TLR ligands as indicated. Peptidoglycan (PGN, *E. coli* 2 µg/ml), a synthetic analogue of double stranded RNA (Poly I:C 25 µg/ml), lipopolysaccharide (*E. coli*, LPS 20ng/ml), flagellin (A from *Salmonella typhimurium*, B from *Bacillus Subtilis*, 1 µg/ml), imiquimod (5 µg/ml), single stranded Poly U complexed with the cationic lipid Lyovec^R^ (ssPolyU 10 µg/ml) were acquired from Invivogen San Diego CA), and unmethylated DNA (CPG 2395 3 µg/ml), was obtained from Coley Pharmaeceuticals, Wellesley, MA).

### Flow cytometric evaluation of T cell populations

Fluorochrome labeled monoclonal antibodies against CD3, CD4, CD8, CD14, CD45RO, CD45RA, CCR7, CD38, CD69 HLA-DR, Ki-67 and labeled Annexin V were purchased from BD Sciences/Pharmingen. Phycoerytherin conjugated antibodies to TLR2 and TLR3 were obtained from eBioscience, (San Diego, CA) and PE conjugated antibody to an intracellular portion of TLR5 was obtained from Imgenex (San Diego, CA). Cells were identified by forward and side scatter characteristics and were analyzed by flow cytometry (LSR-II, Becton Dickinson, San Jose CA). For detection of TLRs 3 and 5 cells were permeabilized before staining with anti-TLR antibodies.

### Cell proliferation and death

PBMCs were suspended in PBS/0.3% BSA and were labeled with 0.01 mM carboxy-fluorescein diacetate, succinimidyl esther (CFSE, Invitrogen ,Oregon, USA) for 10 minutes at 37°C . Cold fetal bovine serum (Gemini Bio-Products, Woodland,CA) was added and cells were incubated for 5 minute on ice. Samples were centrifuged and resuspended in complete medium and stimuli as indicated. Following 7 days of culture, cells were stained for identification of lymphocyte subsets as above; cellular proliferation was monitored by dilution of CFSE dye and apoptotic cells were identified by binding of PE-conjugated Annexin V (BD Biosciences, San Diego,CA).

### Statistical methods

Group means were compared for statistical significance by use of a Wilcoxon rank test and a p-value of 0.05 was considered nominally significant.
